# Deep Learning-Based Ensembling Technique to Classify Alzheimer's Disease Stages Using Functional MRI

**DOI:** 10.1155/2023/6961346

**Published:** 2023-11-03

**Authors:** Taliah Tajammal, Syed Khaldoon Khurshid, Abdul Jaleel, Samyan Qayyum Wahla, Riaz Ahmad Ziar

**Affiliations:** ^1^Department of Computer Science, University of Engineering and Technology, Lahore 54890, Pakistan; ^2^Department of Computer Science (RCET GRW), University of Engineering and Technology, Lahore 52250, Pakistan; ^3^Department of Computer Science, Kardan University, Kabul 1007, Afghanistan

## Abstract

The major issue faced by elderly people in society is the loss of memory, difficulty learning new things, and poor judgment. This is due to damage to brain tissues, which may lead to cognitive impairment and eventually Alzheimer's. Therefore, the detection of such mild cognitive impairment (MCI) becomes important. Usually, this is detected when it is converted into Alzheimer's disease (AD). AD is irreversible and cannot be cured whereas mild cognitive impairment (MCI) can be cured. The goal of this research is to diagnose Alzheimer's patients for timely treatment. For this purpose, functional MRI images from the publicly available dataset are used. Various deep-learning models have been used by the scientific community for the automatic detection of Alzheimer's subjects. These include the binary classification of scans of patients into MCI and AD stages, and limited work is carried out for multiclass classification of Alzheimer's disease up to six different stages. This study is divided into two steps. In the first step, a binary classification of the subject's scan is performed using Custom CNN. The second step involves the use of different deep learning models along with Custom CNN for multiclass classification of a subject's scan into one of the six stages of Alzheimer's disease. The models are evaluated based on different evaluation metrics, and the overall result of the models is improved using the max-voting ensembling technique. The experimental results show that an overall average accuracy of 98.8% is achieved for Alzheimer's stages classification.

## 1. Introduction

The human brain contains about 86 billion neurons, which are responsible for establishing communication and passing information between different parts of the brain [1]. A disorder or malfunction of these neurons causes serious brain diseases. Alzheimer's is a progressive neurodegenerative brain disease that results in the death of neurons. It causes a loss of functionality performed by the brain cells. Alzheimer's is characterized by the deposition of protein layers around the nerve cells. The intertwining of impaired nerve fibers within and outside the brain's nerve cells is the damage associated with the disease. Alzheimer's disease affects the hippocampus area of the brain, and the ventricles of the brain start expanding. These changes are used to detect the early stages of disease [2]. In the human brain, the cerebral cortex is responsible for logic building, thinking, and dealing with social activities. The higher stages of Alzheimer's disease cause shrinkage of the cerebral cortex. Because of this shrinkage, a person becomes dependent on his caregivers [3]. The disorder is inevitably fatal.

The symptoms of Alzheimer's disease can be used to make a diagnosis. However, in some cases, the symptoms of AD remain hidden for about twenty years. Alzheimer's disease has several stages [4], which are as follows: (i) control normal (CN) is the first stage where no symptoms of the disease are shown. (ii) Significant memory concern (SMC) is the next stage, which is characterized by minor memory-related issues that are difficult to detect and are similar to normal age-related problems. (iii) Early mild cognitive impairment (EMCI) stage causes difficulty in arranging items and planning new things. (iv) The distinguishable symptoms of the disease become visible in the fourth stage called mild cognitive impairment (MCI) stage. Here, the patient is having trouble solving simple math-related problems or managing financial tasks. MCI ends with the reduction in the brain gray matter volume [5]. (v) In the late mild cognitive impairment (LMCI) stage, the person experiences problems remembering details. They need help from their guardians to manage their daily tasks. The patients feel difficulty in their surroundings. (vi) In the last stage of Alzheimer's disease (AD), the person becomes unable to interact with his environment. The last stage often results in a patient's death [4]. The conversion from one stage of AD to another depends on the patient's condition. The symptoms appearing at any particular stage may not be the same for multiple patients.

Alzheimer's disease primarily affects people over the age of 65. Alzheimer's disease is a leading cause of death worldwide [6]. Today, Pakistan ranks as the sixth-most Alzheimer's-affected country in the world. The number of Alzheimer's cases in Pakistan is 0.15 million to 0.2 million [7]. The US is one of the countries with the highest number of Alzheimer's cases, which is reported to be 5.8 million. The studies show that Alzheimer's cases in the UK will reach up to 13.8 million by mid-century [8]. Currently, the number of affected people worldwide is 47 million [9]. Worldwide, Alzheimer's cases are predicted to reach up to 131.5 million by the end of 2050 [7]. Since this is a major problem and is affecting a significant percentage of society, it is important to devise ways to detect it as early as possible. While Alzheimer's disease cannot be reversed, patients' progression from the MCI to the AD stage can be slowed. Early diagnosis of AD is, therefore, highly desirable to enhance the quality of life of patients.

The assessment of abnormal brain modifications related to AD has been made easier through neuroimaging. Different approaches use positron emission tomography (PET), computerized tomography scan (CT), structural magnetic resonance imaging (sMRI), electroencephalography (EEG), single positron emission tomography (SPECT) images, brain scans, blood samples, and cerebrospinal fluid (CSF) biomarkers. This research uses functional magnetic resonance imaging (fMRI), which is noninvasive. fMRI is used to measure functional connectivity between different brain parts. fMRI uses blood oxygenation levels to detect changes in response to neural activity in the brain. Being able to detect the effect of the slightest body movement on the brain, fMRI is used in this work [10].

Hongfei Wang et al. proposed the use of a 3D DenseNet network together with ensembling techniques for the classification of the subject's MRI scan into AD, MCI, and CN stages [11]. 3D CNN is used where each CNN layer is directly connected with another subsequent layer to increase the information flow. Then, the result of different 3D dense networks is combined using a probability fusion-based ensembling technique. Binary classification of AD vs. MCI, AD vs. normal, and MCI vs. normal gives an accuracy of 93.61%, 98.83%, and 98.42%, respectively, while the ternary classification of AD vs. MCI vs. normal gives an accuracy of 97.52%. However, the proposed method is not tested for multiclass classification of all the stages of AD. Modupe Odusami et al. propose the use of functional MRI for binary classification of seven stages of AD classification which includes EMCI/LMCI, AD/CN, CN/EMCI, CN/LMCI, EMCI/AD, LMCI/AD, and MCI/EMCI [12]. A modified version of ResNet-18 is used that uses a dropout of 0.2 to avoid overfitting problems. The proposed model works best for the classification of intermediate stages of MCI; however, the classification of AD vs. CN is not very high.

This research work has used the Alzheimer's disease neuroimaging initiative (ADNI) dataset (https://adni.loni.usc.edu/) for training and testing of the setup. We used data from 142 subjects, having a different number of scans in each of the six classes of Alzheimer's disease. The patients' data were chosen to be between the ages of 55 and 65. Data augmentation techniques (such as flipping, rotation, mirroring, and padding) are applied to get different versions of a single image. For fair results, an equal number of samples are taken from each class of the dataset. We employed the VGG-16 as our primary framework and subsequently carried out research using two strategies. Initially, by arbitrarily normalizing the network weights and training the VGG-16 network from scratch, the second method involves employing two transfer learning algorithms while initializing weights from the trained model: (i) by including an additional convolutional layer and adding dropout and (ii) fine-tuning the network's convolutional layers with our dataset.

VGG-16, ResNet-18, AlexNet, Inception v1, and Custom CNN are assembled for multiclass classification of Alzheimer's disease. The results showed that an accuracy of 98.8% was achieved using the max-voting ensembling technique.

The main contributions of this research work are as follows:

1. We presented a Custom CNN model for the multiclass classification of Alzheimer's disease
2. We provide a solution for improving the performance of multiple models for better predicting the performance of multiclass classification problems using the ensembling approach
3. We performed binary classification of 9 different classes (AD/CN, AD/MCI, AD/SMC, AD/EMCI, AD/LMCI, CN/MCI, CN/SMC, CN/EMCI, and CN/LMCI) using Custom CNN network that is trained using VGG-16 weights

The rest of the paper is organized as follows: Section 2 covers the literature review related to this study.  Section 3 covers the materials and methods. It includes a dataset description for the dataset used in this research. It also presents the methodology applied and different deep learning models used, along with Custom CNN on the collected dataset.  Section 4 presents the experimental setup used for this research work along with the results of the work done. Finally, Section 5 concludes the whole work and presents future work.

## 2. Literature Review

Multiclass classification of AD using different deep learning models is the main objective of this research. For the purpose stated, the previous work done in this regard is analyzed by grouping it into two categories: (i) work done using deep learning, transfer learning, and artificial neural network techniques and (ii) work done using machine learning.

### 2.1. Deep Learning and Transfer Learning

The method employed in [13] has used the ResNet-18 architecture for multiclass classification of Alzheimer's stages. The method was tested using resting state fMRI on 138 subjects from a publicly available dataset. A combination of two parallel VGG-16 layers called “Siamese” was proposed in [14]. To get maximum features from a small dataset of 382 subjects, an extra convolutional layer was added to the VGG-16 architecture. The resulting SCNN model was designed to distinguish between the early four classes of dementia. In [5], the authors have used the Xception transfer learning architecture and custom-based CNN architectures for the binary classification of AD and MCI. The method applied has used two different image modalities for result comparison. A transfer learning-based method that utilizes AlexNet architecture to train models was proposed in [15]. It has used both segmented (gray matter, white matter, and cerebrospinal fluid) and unsegmented images from the OASIS dataset for both binary and multiclass classification of the early four stages. A comparison of segmented and unsegmented approaches showed that the latter performed best with an accuracy of 92.8%.

Another method for AD detection has used a random neural network cluster of fMRI images [16]. The presented technique analyzes five different neural networks (backpropagation (BP) NN, Elman NN, PNN, learning vector quantization (LVQ) NN, and competitive NN) and selects Elman NN as the base classifier for feature selection based on accuracy, which is 92.31%. Finally, 23 abnormal regions of the brain were identified using significant features that were extracted through Elman NN. This method is used to differentiate between two classes: healthy control and AD, and it was tested on the ADNI dataset.

### 2.2. Machine Learning Techniques

A method based on graph theory that used both the sMRI and fMRI datasets to generate input features for support vector machines (SVM) was presented in [17]. The target was to identify patients as having MCI that progresses to AD (MCI-C), MCI-NC that did not transform to AD, healthy control, or AD. The results were computed using two feature selection algorithms, namely, SFC (sequential feature collection) and DCA (discriminant correlation analysis), and an accuracy of nearly 56% and 49% is achieved, respectively, on the ADNI dataset, with the limitation that it did not cover all the stages of AD. Bi et al. have used multiple SVMs to distinguish mild cognitive impairment (MCI) from healthy controls (HC) [18]. The human brain was partitioned into ninety “regions of interest” (ROIs) that worked for brain functional connectivity, and a specific template for anatomical automatic labeling (AAL) was used for ROIs. The technique was tested on an ADNI dataset with data from 93 MCI and 105 HC subjects. The researchers proposed the use of both rs-fMRI and graph theory for the binary classification of MCI and HC.

In [19], a technique based on the combination of features was presented for the multiclass classification of AD into three categories, namely, AD, normal individuals, and MCI. Here, the researchers have used the combination of clinical-based features such as the Functional Activities Questionnaire (FAQ), together with textual features such as gray matter (GM), white matter (WM), and cerebrospinal fluid (CSF), to generate a hybrid feature vector, which was then extracted using different feature extraction techniques. The proposed method has produced an accuracy of 79.8% for multiclass classification but does not cover all the stages of AD. Gupta et al. proposed another feature combination technique in [20]. This method uses a combination of the shape and texture of the hippocampal, measurements of cortical thickness, and volumetric measurements to classify three different stages which are AD, MCI, and healthy control. The classification is done using the linear discriminant analysis (LDA) classifier and tested on *T*1-weighted MRI scans from two different datasets (ADNI and AIBL). Recently, another feature fusion technique based on structural MRI was presented in [21]. The given method incorporates three distinct features, namely hippocampal volume (HV), cortical and subcortical segmented areas, and voxel-based morphometry (VBM), into one feature for the classification of 326 subjects. It is trained to distinguish healthy individuals from AD patients and MCI subjects.

Recent work done in this field includes the detection of the early stages of Alzheimer's disease. The models have been designed to predict the difference between normal individuals (called “healthy controls”) and patients with AD (Alzheimer's disease) or to classify multiple stages. Most of the time, the classification is done using structural MRI or PET imaging. AD classification using fMRI is limited. As fMRI scans provide massive information about brain structure and capture the resting state of the brain as well as provide the cognitive details that are helpful for AD classification, this study used functional magnetic resonance imaging (fMRI) to classify Alzheimer's disease.

## 3. Materials and Methods

### 3.1. Dataset Description

In this research, the Alzheimer's disease neuroimaging initiative (ADNI) dataset (https://adni.loni.usc.edu/) is used as it provides good-quality images. ADNI is a famous neuroimaging study. ADNI encourages researchers to perform comprehensive analyses with its generic dataset and exchange valid results with other researchers throughout the world. This work used data from 142 subjects, with a different number of scans in each of the six classes. The data of patients aged 55 to 65 are selected.  Table 1 contains a detailed description of the subjects. The dataset contains images from three different views, which are axial, coronal, and sagittal.  Figure 1 shows a sample image from the ADNI dataset.

### 3.2. Methodology

The methodology applied in this study uses a pipeline of medical imaging processing for the classification of the input image. The first step is to preprocess the dataset to eliminate anomalies and noise, and to make the entire dataset uniform. The next step is to perform classification by extracting features using a Custom CNN. In this study, we performed both binary and multiclass classifications of AD. Using Custom CNN, a subject's scan is classified into one of the following classes: AD vs. CN, MCI vs. AD, CN vs. MCI, AD vs. SMC, EMCI vs. AD, LMCI vs. AD, CN vs. SMC, EMCI vs. CN, LMCI vs. CN. Different CNN models are used for multiclass classification, along with Custom CNN. The results of different models for multiclass classification of AD into one of the six possible stages are then ensembled.  Figure 2 depicts the detailed methodology process.

#### 3.2.1. Preprocessing Techniques

A preprocessing pipeline consisting of standardized methods is used for this study. Preprocessing techniques are divided into a number of steps that are sequential in nature. The dataset used contains fMRI scans in a nifty format. This work uses the Functional Magnetic Resonance Imaging of the Brain (FMRIB) Software Library (FSL).

(1) Reorientation. In the first step, the files are reoriented. Reorientation is done so that all the images are displayed in the same way when viewed. This includes 90°, 180°, and 270° rotation of images about different axes.
(2) Skull Stripping. Skull stripping is performed to remove cranial or bony parts from scans, including the eyes and neck tissues. This is done using FSL-BET, which works on the basis of an intensity value that lies between 0 and 1 as shown in equation (1). Here, *I* is the input image on which the function *f* of FSL-BET is applied. Thresholding is used to separate dark pixels (background skulls and cavities) from bright pixels (brain, skin, eyeballs, and facial tissues).
  (1) $$\begin{array}{c} \text{Skull stripped image}=\left\{\begin{array}{c} 0\leq f\left(I_{x,y,z}\right)\leq 0.5---brain\;t\text{issues},\\ 0.5\leq f\left(I_{x,y,z}\right)\leq 1---s\text{kull}. \end{array}\right. \end{array}$$
(3) Motion Correction. One of the major problems during fMRI data collection is the participant's motion, which includes shaking the head left or right. This badly affects the quality of the data collected. To reduce the effect of the subject's motion, motion correction is performed using FSL-MCFLIRT. It is done by selecting a reference image from the series of all the images and registering each image in turn to this fixed reference.
(4) Slice Timing Correction. The fMRI image consists of different slices taken at different moments. 3D brain volume images can be obtained by stacking 2D slice images anywhere from a fraction of a second to several seconds, depending upon the number of slices and their resolution. There are delays during these slice stackings. Slice timing correction is used to correct these delays by temporally aligning all the slices with reference to a time point. To overcome this difference in slice timings, the FEAT module of FSL is used. Here, interpolation is used for the temporal adjustment of voxels and to estimate a single value between the sample points.
(5) Spatial Smoothing and Normalization. To decrease the noise level while retaining the underlying signal, spatial smoothing is applied. During this technique, each voxel's intensity is calculated as a weighted average of its intensity and its near points within a set radius. Spatial smoothing is performed using the FWHM Gaussian kernel of size 6 mm.
In order to remove the noise and psychological artifacts introduced due to the subject's motion (such as breathing and heartbeat), temporal high pass filtering is used with a frequency of 0.01. For spatial normalization, the images are registered according to the reference template of 152 MRI scans, which is the MNI-152 template. This is done by applying a linear transformation to images using 12 degrees of freedom (DOF). This task is performed using the FSL FLIRT module.
(6) Histogram Equalization. Histogram equalization is done to enhance the contrast of images. However, this method is suitable when the image has a nearly similar distribution of pixel values. In this study, different MRI scans are used, and the scans have varying pixel distribution values.
(7) Contrast Limited Adaptive Histogram Equalization. This technique is used to obtain high-quality and clear images. This technique works by creating separate histograms for different regions of an image. In this work, the image is divided into a grid of size 8 × 8, and equalization is applied to each pixel of the grid. By the hit and trial method, the clip limit is set to 2.0 for better contrast.
(8) 3D to 2D conversion. The above-mentioned preprocessing steps result in 64 × 64 × 48 × 140 fMRI scans, with each scan including 64 × 64 3D-48 volumes per scan (a total of 140 scans). On average, one fMRI scan contains about 48 volumes, which results in 48 slices for each fMRI. The first and last 10 slices are removed for each scan as they contain no functional information and are just black. Each slice is then converted into 2D along the image height and time axis. This is useful as neural networks work well with 2D images.  Figure 3 shows the process by which each slice of an image is saved as a separate layer in PNG format.

To get good classification results, a balanced dataset is necessary. Data augmentation techniques such as flipping, rotation, mirroring, and padding are applied to get different versions of a single image. For fair results, an equal number of samples are taken from each class of the dataset. The total number of images acquired for each class before and after data augmentation is shown in Table 2.

#### 3.2.2. Classification Stage

Different deep-learning models are used for classification. The input image is of size 64 × 64 and is in grayscale for all the models, which are described as follows:

1. VGG-16. Visual geometry group, or VGG, is the famous convolutional neural network that has different types of layers, which include convolutional layers, pooling layers, and fully connected layers. The inclusion of features in an input image is defined by convolutional layers. To get the exact features of the input image, the downsampling of feature maps is done using pooling layers. The pooling layer works independently on each function map to construct a new collection of the same number of pooled function maps. We have used VGG-16, which has 16 layers in total. The network is composed of a stack of 13 convolutional layers with three fully connected layers. It uses a filter of size 3 × 3 in each convolutional layer with stride 1 and an activation function called rectified linear unit (relu). To reduce the feature maps, max pooling is performed on few convolutional layers with pool size 2 × 2 and stride 2. The results are then flattened and passed through two fully connected layers having 4096 channels each, followed by a softmax activation layer having six output neurons for six different classes. The detailed architecture of the VGG-16 model used for Alzheimer's classification is shown in Figure 4.
2. ResNet-18. As the network starts increasing in depth, there exists a problem of accuracy degradation or vanishing gradient. To solve this problem, ResNet-18 was introduced. It differs in the sense that it uses skip connectors to connect the output of the previous layer to the next layer. Similarly, the network can anticipate which feature it was studying before with the feedback applied to it if we skip the input to the first layer of the model to be the output of the last layer of the model. In general, the inputs are skipped after every two convolutions. We have trained the model using ResNet-18, which has 17 convolutional layers and 1 fully connected layer. The network uses a kernel of size 3 × 3 with stride 1. The layers work with the same filter size as long as the output feature maps have the same dimensions and are doubled by halving the output feature map. The output of layers is passed to the average pooling layer with pool size 8, followed by a flattening layer that flattens the results.  Figure 5 shows the architecture diagram of ResNet-18 used for the classification of Alzheimer's disease.
3. Alex Net. This network uses 8 layers, including 5 convolutional layers and 3 dense layers. It has the ability to multi-GPU train by allowing half of the neurons to be trained on another GPU. The addition of dropout and LRN (local response normalization) distinguishes this network. The architecture of the model used for Alzheimer's classification is provided in Figure 6. The input image is convolved with 96 filters of size 11 × 11 followed by a max pooling layer of pool size 2 × 2. Similarly, in the second convolutional layer, 256 filters of size 5 × 5 are convolved with 32 × 32 input images. Each convolutional layer is followed by a max pooling layer except the last two, which are stacked. In AlexNet, the neurons of one layer are connected to all the neurons of the next layer via three dense layers, as shown in Figure 6. Finally, the output is classified using the softmax function, which sums the probability of all outcomes to 1.
4. Inception v1/GoogLeNet. Inception v1 or GoogLeNet differs in that it broadens rather than deepens the network and is characterized as “sparse” architecture. Instead of having the same filter size, it works by having a different-sized kernel that operates on the same level. Here, convolution is performed with 1 × 1, 3 × 3, and 5 × 5 filters with max pooling using ×3 and stride 1. The output of all filters is then concatenated for the next layer.  Figure 7(a) shows the naive version of inception. To reduce the computational cost of the network, the images are convolved with 1 × 1 filters before convolving with other filters. This helps reduce the dimensions of feature maps.  Figure 7(b) shows the Inception architecture of the model for dimensionality reduction.
5. Custom CNN. A CNN-based approach inspired by VGG-16 called “Custom CNN” is developed. It is designed using one additional convolutional layer to obtain maximum features from the training samples. It is similar to VGG-16 but has 14 convolutional layers and 5 max pooling layers. The network uses filters of size 3 × 3 with pool size 2. The network uses a dropout of 0.2 and a fine-tuning approach in which more than one layer of the network is retrained from the samples of the new task. For a fine-tuning approach, we retrained all the convolutional layers of the network with our dataset. In this approach, we used the weights of the VGG-16 network as the base point for fine-tuning the layers.  Figure 8 shows the architecture of the Custom CNN used for Alzheimer's disease classification.

#### 3.2.3. Ensemble

Ensembling is used to reduce the variance involved in deep learning models for predicting the output of Alzheimer's stage classification. During the training phase, the model learns a distinct set of weights, which in turn produce different outputs. To overcome this variation in output, several models are trained, and the results are combined for the final prediction. Different methods of ensembling are used for this research work, which are as follows:

1. Stacking. In this technique, the output of multiple models is used to build a new model, which is then used for final output classification. This method operates by enabling a training algorithm to ensemble multiple similar learning algorithms' predictions. It involves the use of the complete training dataset for predicting the model output. This research uses different deep learning models (discussed above) as the base models and uses the predictions of these models to create further layers of models. The results of these layers are then combined to produce the final result.
2. Blending. This technique is similar to stacking, with the difference that the complete training data is not used for training the base model. Instead, a small portion of training data is used for training the base model, and test data are used for making predictions.
3. Averaging. In the averaging method, several predictions are made for each class by the models, and the final outcome is calculated by finding the average of the model outcomes.
4. Max Voting. This technique uses the count of the maximum vote made by each model for the predicted class. Each base model predicts and votes for each sample during max voting. The final prediction class only contains the sample class with the most votes. In this study, the output of all the deep learning models used is finalized using the max-voting technique.

For Alzheimer's disease classification, ensembling of VGG-16, ResNet-18, AlexNet, Inception V1, and Custom CNN is performed as shown in Figure 9. Ensembling of different models used for AD classification is tested for stacking, blending, averaging, and max voting. The outcomes are presented in the next section and evaluated on the basis of well-known metrics.

## 4. Results and Discussion

This work aims to classify Alzheimer's patients into one of the six stages by training different models. For this purpose, we trained VGG-16, ResNet-18, AlexNet, Inception V1, and Custom CNN on the ADNI dataset. A layer-wise outcome for VGG-16 execution on the ADNI dataset is shown in Figure 10.

The performance of the trained models is evaluated using different evaluation metrics, for which the following terms are used:

  True Positive (TP). The number of cases where the model predicts the stage of Alzheimer's disease correctly and it is true in actuality.
  False Positive (FP). The number of cases where the stage of Alzheimer's disease that the model predicts is not real in actuality.
  True Negative (TN). The number of cases in which the model predicted that a specific Alzheimer's stage was invalid and that stage was, in fact, invalid.
  False Negative (FN). The number of cases in which the model predicted that a specific Alzheimer's stage was invalid but that stage was actually valid.

In the context of the above-described values, different evaluation metrics used for Alzheimer's disease classification are as follows:

Accuracy. Accuracy is the measure of how accurately the model predicts various stages of Alzheimer's and is defined as follows:
  (2) $$\begin{array}{c} \text{Accuracy}\left(A\right)=\frac{\text{True}\text{ positive}+\text{true}\text{ negative}}{\text{Number of}\text{ samples}\text{ in ADNI dataset}}. \end{array}$$
Recall/Sensitivity/True Positive Rate. Out of all the Alzheimer's stages that the models predict (positive cases), this is a measure of how much the model correctly predicts the stage.
  (3) $$\begin{array}{c} \text{Recall}\left(R\right)=\frac{\text{True positive}}{\text{True}\text{ positive}+\text{false}\text{ negative}}. \end{array}$$
Precision. For all the Alzheimer's stages predicted correctly (positive cases), it defines how many Alzheimer's stages are true.
  (4) $$\begin{array}{c} \text{Precision}\left(P\right)=\frac{\text{True positive}}{\text{True positive}+\text{false}\text{ positive}}. \end{array}$$
Specificity/True Negative Rate. Out of all the negative classes predicted correctly, it defines how many cases are predicted correctly by the model.
  (5) $$\begin{array}{c} \text{Specificity}\left(S\right)=\frac{\text{True negative}}{\text{True}\text{ negative}+\text{false}\text{ positive}}. \end{array}$$
*F*1 Score. It is the average of precision and recall.

(6) $$\begin{array}{c} F1\text{ score}=\frac{2\times \left(\text{precision}\times \text{recall}\right)}{\text{recall}+\text{precision}}. \end{array}$$

### 4.1. Binary Classification Results

Table 3 displays the binary classification of the subject's scan for nine different groups: AD vs. CN, MCI vs. AD, CN vs. MCI, AD vs. SMC, EMCI vs. AD, LMCI vs. AD, CN vs. SMC, EMCI vs. CN, and LMCI vs. CN. Custom CNN was used to achieve these results.

The result of the binary classification of different stages shows that our Custom CNN was able to classify the AD vs. CN stages with a high accuracy of 99.6%. This is due to the fact that there are great visible differences between the subject's scans for these two classes. Similarly, MCI and AD are two prominent classes that have significant structural and functional variations. The Custom CNN model was able to get maximum features from these two classes of the dataset and was thus able to obtain an accuracy of 99.4%. A comparison of control normal and healthy individuals with MCI stage reveals that the model accurately classified MCI patients up to 99.8% of the time. For other intermediate classes such as SMC, EMCI, and LMCI, their binary classification accuracy is not as high as that of classes such as CN, MCI, and AD.

### 4.2. Multiclass Classification Results

The comparison results of different models for predicting Alzheimer's disease stage are shown in Table 4. The performance metrics for several different image classification models are found as follows. VGG-16 has an accuracy of 96.2%, precision of 91.4%, recall of 89.9%, specificity of 90.4%, and *F*1 score of 93.7%. ResNet-18 has an accuracy of 87.5%, precision of 85.4%, recall of 88.6%, specificity of 84.3%, and *F*1 score of 86.5%. AlexNet has an accuracy of 91.4%, precision of 88.5%, recall of 86.5%, specificity of 84.8%, and *F*1 score of 85.8%. Inception v1 has an accuracy of 88.6%, precision of 89.3%, recall of 90.3%, specificity of 88.2%, and *F*1 score of 90.1%. Custom CNN has an accuracy of 96.2%, precision of 91.4%, recall of 94.8%, specificity of 93.6%, and *F*1 score of 95.3%. In general, higher accuracy, precision, recall, and *F*1 score indicate better performance of the model. Results show that Custom CNN performs better among all the models for the underlying problem due to better training of weights for this particular dataset. The results of all the models are ensembled using the max-voting technique, which produces an overall accuracy of 98.8% for Alzheimer's disease stage classification.

Figure 11 shows the comparison of different models based on loss and accuracy. The main target is to reduce the loss while obtaining maximum accuracy. The graphs of various models show that accuracy generally increases with increasing epochs and loss decreases. Small fluctuations are because models continue to learn about the exact features of the training set. The models produce random guesses about disease stage prediction.

Next, we have used the ensemble technique to make final predictions. We present the results for stacking blending, averaging, and max-voting-based predictions as shown in Table 5. For the underlying problem, the results show that an accuracy of 94.3% is achieved with stacking, 92.5% with blending, and 97.9% with averaging and 98.8% accuracy is achieved using the max voting. Hence, the best results are achieved with the max-voting-based ensembling technique for Alzheimer's disease.

### 4.3. Comparison with State-of-the-Art Research Work

In this research work, two different approaches are adopted. In the first step, binary classification is performed. We divided the AD stages into nine groups as given in Table 3. For multiclass classification of the subject's scan into one of six possible stages, an ensembling approach is used.

Table 6 shows the comparison of existing work done for Alzheimer's disease classification that has used an ensembling approach. A deep learning-based ensembling technique was presented by Loddo [22]. This study performed a four-class classification of dementia stages using the AlexNet, ResNet-101, and Inception ResNetV2 models on several different datasets. The average ensembling technique was used on each selected dataset, and the maximum overall accuracy achieved was 98.24%.

Another study presented the use of deep learning models for AD classification [23]. They used AdaBoost as an ensembling technique for merging the results of GoogleNet, ResNet, and DenseNet. The technique was able to perform binary classification of the AD vs. HC and MCI vs. HC stages with an overall accuracy of 93%. Similarly, a three-stage classification of AD into AD vs. MCI vs. CN stage using several DenseNet models was performed in [11] that used the probability fusion method for ensembling purposes, and the maximum accuracy for three class classifications using this approach was 97.52%. Karwath et al. have used the majority voting technique for predicting the best outcome of different classifiers [24] which performed a binary classification of AD vs. healthy and mild MCI vs. severe MCI with an accuracy of 91% and 85%, respectively. The proposed work in this study uses different deep learning models, and the results of these models are then ensembled using different techniques, out of which the max-voting technique has performed best. Previous work done in this field includes ensembling approaches for less than six-stage classification. To our knowledge, this is the only study that has used the ensembling technique for the six-stage classification of AD.

## 5. Conclusion and Future Work

Using fMRI scans, this study presented a technique for categorizing Alzheimer's disease into six stages. The Alzheimer's disease neuroimaging initiative (ADNI) dataset has been used for training the classifier on fMRI images of the patients to identify the six stages of Alzheimer's disease. The data of patients aged 55 to 65 are chosen, and data augmentation techniques are applied to obtain different versions of a single image. An equal number of samples are drawn from each dataset class to ensure fair results. There are nine different groups of AD stages, and binary classification with Custom CNN is applied to classify scans of subjects into one stage. For multiclass classification of AD, the results of VGG-16, ResNet-18, AlexNet, Inception V1, and Custom CNN are combined. The results show that the max-vote ensembling technique achieves 98.8% accuracy. As deep learning models are expected to bring breakthroughs for medical image diagnosis, the techniques used in this paper can be cross-validated using another neuroimaging dataset. The work can be extended by increasing the dataset and validating it using recurrent neural networks. Furthermore, report generation functionality can be added, which makes it easy for the common man to read and understand the reports.

## Figures and Tables

**Figure 1:** Sample image from ADNI dataset. (a) Axial view. (b) Coronal view. (c) Sagittal view.

**Figure 2:** Architecture diagram of the methodology used for AD classification.

**Figure 3:** 3D to 2D conversion process.

**Figure 4:** VGG-16 architecture used for AD classification.

**Figure 5:** ResNet-18 architecture used for AD classification.

**Figure 6:** AlexNet architecture used for AD classification.

**Figure 7:** (a) Naive version of Inception. (b) Inception architecture.

**Figure 8:** Custom CNN architecture used for AD classification.

**Figure 9:** Ensembling of different models used for AD classification.

**Figure 10:** VGG-16 execution on ADNI dataset.

**Figure 11:** Loss and accuracy graph of different models used for AD classification.

**Table 1:** Description of the dataset used for AD classification.

Class	Subjects	fMRI	Male	Female	Age
AD	24	1,566	20	4	55–57
CN	24	1,376	20	4	56-57
EMCI	24	1,471	12	12	56–58
MCI	24	1,260	2	22	56–58
LMCI	22	856	12	12	55–57
SMC	24	1,183	9	15	63–65
Total	**142**	**7,712**			

The bold values show the total count of subjects taken and the respective number of fMRI images for performing the experiment in this research work.

**Table 2:** Dataset description before and after preprocessing.

Class	Before augmentation	After augmentation
AD	50,101	1,35,000
CN	52,518	1,35,000
EMCI	49,552	1,35,000
MCI	47,856	1,35,000
LMCI	44,840	1,35,000
SMC	45,420	1,35,000
Total	**2,90,287**	**8,10,000**

The bold values show the count of images before and after applying data augmentation techniques.

**Table 3:** Evaluation metrics results of different models on the ADNI dataset.

Group	Accuracy (%)	Precision (%)	Recall (%)
AD vs. CN	99.6	94.3	95.8
MCI vs. AD	99.4	96.2	96.6
CN vs. MCI	99.8	94.5	95.7
AD vs. SMC	93.4	90.6	92.6
EMCI vs. AD	93.5	91.4	94.5
LMCI vs. AD	91.3	89.7	90.2
CN vs. SMC	92.4	90.5	93.4
EMCI vs. CN	93.2	92.3	89.7
LMCI vs. CN	92.5	90.5	89.6

**Table 4:** Evaluation metrics results of different models on the ADNI dataset.

Models	Accuracy (%)	Precision (%)	Recall (%)	Specificity (%)	*F*1 score (%)
VGG-16	96.2	91.4	89.9	90.4	93.7
ResNet-18	87.5	85.4	88.6	84.3	86.5
AlexNet	91.4	88.5	86.5	84.8	85.8
Inception v1	88.6	89.3	90.3	88.2	90.1
Custom CNN	96.2	91.4	94.8	93.6	95.3

**Table 5:** Comparison results of different ensembling techniques.

	Stacking (%)	Blending (%)	Averaging (%)	Max voting (%)
Accuracy	94.2	92.5	97.9	98.8

**Table 6:** Comparison of state of the methods for AD classification.

Study	Year	Stages	Method	Ensembling technique	Accuracy
Loddo et al. [22]	2022	NC/VM-AD/Mi-AD/Mo-AD	AlexNet, ResNet-101, and Inception ResNetV2	Averaging	98.24%
Fang et al. [23]	2020	AD/HC, MCI/HC	GoogleNet, ResNet, and DenseNet	AdaBoost	93%
Wang et al. [11]	2020	AD/MCI/CN	DenseNet	Probability-based fusion	97.52%
Karwath et al. [24]	2017	AD/healthy, mild MCI/severe MCI	Alexnet CNN	Majority voting	AD/Healthy => 91%, Mild MCI/severe MCI => 85%
This study	2022	AD/SMC/EMCI/MCI/LMCI/CN	VGG-16, ResNet-18, Inception V1, AlexNet, and Custom CNN	Max voting	98.8%

## Data Availability

Data are available upon request.
